# Effects of Roflumilast on Patients with Chronic Obstructive Pulmonary Disease Treated with Inhaled Corticosteroid/Long-Acting *β*2 Agonist: A Meta-analysis

**DOI:** 10.1155/2022/8101099

**Published:** 2022-07-23

**Authors:** Shasha Zeng, Haibing Bai, Mi Zou

**Affiliations:** ^1^Department of Internal Medicine, Chongqing Nanan Traditional Chinese Medicine Hospital, Chongqing 400060, China; ^2^Respiratory Department, The First Branch of the First Affiliated Hospital of Chongqing Medical University, Chongqing 400015, China

## Abstract

**Objective:**

Roflumilast is a novel therapeutic drug for chronic obstructive pulmonary disease (COPD). This study was designed to evaluate the efficacy and safety of roflumilast combining inhaled corticosteroid (ICS)/long-acting *β*2 agonist (LABA) in treating COPD patients through the meta-analysis.

**Methods:**

Randomized controlled trials of roflumilast combining ICS/LABA in treating patients with severe and profound COPD were searched from PubMed, Cochrane Library, and Embase databases from their establishment to February 2022. The quality of included studies was assessed by Cochrane risk bias assessment tool. The main outcomes of these studies should include at least one of the following clinical outcome indicators: forced expiratory volume in one second (FEV_1_), exacerbation rate, and adverse events (AEs) such as diarrhea, nasopharyngitis, and headache.

**Results:**

Six articles were included in the study, including 9,715 patients. Meta-analysis revealed that compared with placebo, roflumilast gained superiority for severe COPD patients treated with ICS/LABA combinations in FEV_1_ before bronchodilator administration (MD = 46.62, 95% CI (30.69, 62.55), *P* < 0.00001), FEV_1_ after bronchodilator administration (MD = 45.62, 95% CI (34.95, 56.28), *P* < 0.00001), and COPD exacerbation rate (RR = 0.90, 95% CI (0.87, 0.94), *P* = 0.001). In terms of safety, the incidence of diarrhea, headache, nausea, weight loss, back pain, loss of appetite, and insomnia was notably higher in the roflumilast group than in the placebo group.

**Conclusion:**

Roflumilast is suggested to be significantly effective for severe COPD patients with ICS/LABA combination therapy, which reduces the exacerbation rate but also leads to PDE4 inhibitor-related adverse reactions.

## 1. Introduction

Chronic obstructive pulmonary disease (COPD) is a chronic respiratory disease with a high risk of death, and its incidence is high among smokers, which gradually increases with age [1]. The obstruction often occurs in small airways with diameter < 2 mm in COPD patients, resulting in airflow limitation. After bronchodilator administration, the decrease of patient's forced expiratory volume in one second (FEV_1_) can reflect airflow limitation and lung functions, which can be utilized to diagnose the disease severity of COPD patients [2, 3]. Increased airflow limitation in COPD patients may increase the exacerbation risk of symptoms, and this limitation possesses incomplete reversibility, whereas bronchodilators relax airway smooth muscle and increase tension, making it relatively reversible [4]. Furthermore, inflammation in the lungs or the whole body would have occurred in patients with COPD exacerbation, while inhaled corticosteroid (ICS) can reduce the exacerbation rate of COPD by arresting inflammation [5]. A clinical trial revealed that ICS combining dual bronchodilators is effective for patients with severe COPD at high exacerbation risk [6]. However, the treatment of COPD has been gradually relying on the combination therapy of ICS and long-acting bronchodilators in recent years, which may have safety risks or limit the disease control and prevention management of COPD [7]. Therefore, drugs that are more suitable for treating severe COPD or that can be used in combination with ICS to increase the treatment efficiency are continuously required.

Roflumilast is a phosphodiesterase-4 inhibitors (PDE4), which has anti-inflammatory effects and can inhibit the release of inflammatory mediators, thus advantageously treating the respiratory diseases, such as pulmonary inflammation complicated by asthma and COPD [8]. In terms of treating severe to profound COPD, roflumilast could attenuate frequent exacerbation of symptoms in patients, thus enabling them enter a stable period and reducing the history of exacerbation and the times of hospitalization [9, 10]. Meanwhile, roflumilast is well tolerated and has a favorable affinity with phosphodiesterase 4, which could effectively ameliorate lung functions of patients with severe to profound COPD [8, 11]. Nowadays, roflumilast generally functions as an adjunct to combination therapy of ICS and long-acting bronchodilators to further improve the drug efficacy in patients with severe to profound COPD. Long-acting beta2-agonists (LABAs) and long-acting muscarinic antagonists (LAMAs) are the widely used bronchodilators in combination therapies for severe COPD [12]. Roflumilast combining LABA/LAMA was pointed out to ameliorate lung functions of COPD patients, which is more effective than those treated with LABA or LAMA alone. Besides, roflumilast combining ICS/LABA or ICS/LABA/LAMA can effectively reduce the exacerbation rate of COPD [10, 13].

Therefore, we conducted a meta-analysis to comprehensively evaluate the efficacy and safety of roflumilast combining ICS/LABA or ICS/LABA/LAMA in patients with severe COPD.

## 2. Methods

### 2.1. Literature Retrieval

Randomized controlled trials (RCTs) of roflumilast combining ICS/LABA in COPD patients were retrieved from PubMed, Cochrane library, and Embase databases. All related English literature was researched from the establishment of databases to February 2020, whose keywords consisted of “roflumilast”, “inhaled corticosteroid”, “long-acting *β*2 agonist”, and “chronic obstructive pulmonary disease”.

### 2.2. Selection of Literature

#### 2.2.1. Inclusion Criteria

(1) Subjects: patients diagnosed with severe COPD by histopathological examination. At the same time, their spirometry showed airflow obstruction (after passing bronchodilator, forced expiratory volume in one second and forced vital capacity (FEV_1_/FVC) < 0.70); (2) study type: phase III/IV RCTs; (3) interventions: combination treatment of roflumilast and ICS/LABA for COPD; (4) control group: combination treatment of placebo and ICS/LABA for COPD; and (5) outcome indicators: the following descriptions were included: FEV_1_, exacerbation rate, and AEs (such as diarrhea, nasopharyngitis, and headache).

#### 2.2.2. Exclusion Criteria

(1) The intervention contained only ICS or LABA, or the control drug was not a placebo; (2) animal experiments; (3) non-English literature, repeatedly published literature, or guidelines, review, case analysis, expert experience, meeting records, technical reports, and editorials; (4) literature with inconsistent data or could not be extracted; and (5) therapeutic drugs mentioned in the literature were not approved by the drug administration.

### 2.3. Data Extraction and Quality Assessment

Two investigators extracted the data independently, and a third investigator mended their divergences. These data, including author, year of publication, trial stage, sample size, interventions, FEV_1_, exacerbation rate, and AEs, were extracted from the trials. Quality assessment of the included studies was performed employing Cochrane bias risk assessment tool. This scale mainly evaluated the bias risk with 7 items in 6 aspects, including random sequence generation, allocation concealment, blind evaluation of investigators and subjects, blind evaluation of outcomes, integration of outcome data, reporting bias, and other obvious biases. The results of “low-risk bias,” “high-risk bias,” and “unclear” were obtained.

### 2.4. Statistical Methods

The Review Manager 5.4 software was applied for meta-analysis. Risk ratio (RR) served as the effect index for the count (dichotomous) data, and mean difference (MD) was utilized as the effect index for measurement (continuous variable) data, with point estimate values and 95% confidence intervals (CI) given for each effect size. The heterogeneity among results was determined by chi-square test, and the size of heterogeneity was quantitatively determined by combining *I*^2^. *I*^2^ ≤ 50% and *P* ≥ 0.1 were considered to indicate no statistical heterogeneity among studies, and a fixed-effect model was carried out. Otherwise, heterogeneity was considered, and a random-effect model was applied for meta-analysis.

## 3. Results

### 3.1. Literature Retrieval Results

136 studies were discarded in the 146 preliminarily searched literature by browsing titles and abstracts (guidelines, review, case analysis, expert experience, meeting records, technical reports, editorials, and republications). Among the 10 remaining literature, 4 were excluded after a full-text review, and other 6 studies [10, 14–18] that met the criteria were included.  Figure 1 displays the literature screening process.

### 3.2. Basic Features and Quality Assessments of the Included Literature

Finally, 9,715 COPD cases were enrolled in the 6 included literature. Among them, 5,045 patients were treated with roflumilast combining ICS/LABA, and 4,670 patients were treated with placebo combining ICS/LABA. In 3 involved literatures [15–17], some patients were dosed with short-acting *β*2 receptor agonist (SABAs) during the trial according to the actual situation. In all included treatment methods, patients were treated with or without LAMAs in line with their actual situation. The basic features of the included studies are indicated in Table 1. Cochrane bias risk assessment revealed that, except the large bias caused by the withdrawal of more cases from the trial due to adverse reactions in the experimental group than in the control group, other kinds of bias risk were at a low level. The overall quality of the included literature was relatively high, as represented in Figures 2(a) and 2(b).

### 3.3. Meta-analysis Results

#### 3.3.1. Changes in FEV_1_ before Bronchodilator Administration Relative to Baseline

Four studies were included. FEV_1_ was evidently increased in the roflumilast group before bronchodilator administration, whereas FEV_1_ decrease was observed in the placebo group. Meta-analysis of the random-effect model illustrated that the difference between experimental group and control group was significant when *α* = 0.05 (MD = 46.62, 95% CI (30.69, 62.55), *P* < 0.00001), as shown in Figure 3.

#### 3.3.2. Changes in FEV_1_ after Bronchodilator Administration Relative to Baseline

Four studies were included. FEV_1_ was notably increased in the roflumilast group after bronchodilator administration, whereas FEV_1_ decrease was observed in the placebo group. Meta-analysis of the random-effect model illustrated that the difference between experimental group and control group was significant when *α* = 0.05 (MD = 45.62, 95% CI (34.95, 56.28), *P* < 0.00001), as exhibited in Figure 4.

#### 3.3.3. COPD Exacerbation

Three studies were eventually included for exploring COPD exacerbation. The results of meta-analysis demonstrated that COPD exacerbation rate in the roflumilast group was remarkably lower than that in the placebo group, and the difference was statistically significant (RR = 0.90, 95% CI (0.87, 0.94), *P* = 0.001), as displayed in Figure 5.

#### 3.3.4. Adverse Reactions

Among the adverse reactions, each of diarrhea, headache, nausea, and nasopharyngitis was included in 4 literatures. Each of weight loss, appetite loss, insomnia, back pain, influenza, pneumonia, hypertension, and death was included in 3 literature, and upper respiratory tract infection was included in 2 literatures. Meta-analysis of the fixed-effect model confirmed that the incidence of diarrhea (RR = 2.95, 95% CI (2.45, 3.56), *P* < 0.00001), headache (RR = 1.95, 95% CI (1.56, 2.43), *P* < 0.00001), nausea (RR = 2.58, 95% CI (2.01, 3.30), *P* < 0.00001), weight loss (RR = 3.41, 95% CI (2.74, 4.24), *P* < 0.00001), appetite loss (RR = 5.01, 95% CI (3.18, 7.90), *P* < 0.00001), insomnia (RR = 2.17, 95% CI (1.58, 2.96), *P* < 0.00001), and back pain (RR = 1.45, 95% CI (1.09, 1.94), *P* = 0.01) was markedly higher than that in the placebo group, and the differences were statistically significant, as presented in Figure 6.

As indicated in Figure 7, there was no statistically significant difference in incidence of nasopharyngitis (RR = 0.93, 95% CI (0.78, 1.10), *P* = 0.39), influenza (RR = 1.08, 95% CI (0.83, 1.41), *P* = 0.58), pneumonia (RR = 1.02, 95% CI (0.82, 1.28), *P* = 0.85), upper respiratory tract infection (RR = 0.88, 95% CI (0.68, 1.12), *P* = 0.30), hypertension (RR = 0.81, 95% CI (0.62, 1.05), *P* = 0.12), and death (RR = 1.05, 95% CI (0.78, 1.41), *P* = 0.74) between the roflumilast group and placebo group.

## 4. Discussion

COPD exacerbation is an acute event characterized by worsening of respiratory symptoms, which requires alterations of drug therapy and/or hospitalization [19]. Therefore, drug therapy for COPD is designed to relieve symptoms and reduce the risk of AEs such as exacerbation, disease progression, and death [20]. The combination of ICS/LABA has been shown to reduce acute exacerbations of COPD and is often the preferred treatment for COPD [21, 22]. However, acute exacerbations of COPD are usually associated with high level of inflammation in the body [23]. Roflumilast can reduce the levels of inflammatory markers in the airway of COPD patients and is approved for long-term treatment in combination with ICS and long-acting bronchodilators of patients at high risk of acute exacerbation [24]. As roflumilast is recommended as an adjunct agent for patients with severe COPD, its combination with ICS/LABA effectively decreases the exacerbation risk in patients with severe COPD [25]. This study evaluated the efficacy and safety of roflumilast in patients with moderate to severe COPD using RCT data in combination with inhaled ICS/LABA.

The results suggested that compared with placebo, roflumilast remarkably ameliorated lung functions (as measured with FEV_1_ before and after bronchodilator administration) and reduced the incidence of COPD exacerbation in patients with moderate to severe COPD. FEV_1_ improvement plays a crucial role in determining the efficacy of new drugs for COPD [20]. In one included study, the end-point values of FEV_1_ before and after bronchodilator administration are higher in the roflumilast group than the baseline level, while FEV_1_ reduction was observed in the placebo group, which is in line with previous studies [26].

Heterogeneity is attributed to the differential definition of COPD exacerbation. In 3 literatures including this index, moderate to severe exacerbation is defined as the need for oral or parenteral glucocorticoid therapy (with or without antibiotics) and being hospitalized, or dead, or both. As a previous study described, roflumilast and ICS may reduce inflammation through different mechanisms. The combination of these agents may be cumulative or synergistic, and the utilization of their combination may provide clinical benefits beyond those achieved by single ICS, single PDE4 inhibitor, or ICS/LABA combination therapy [27]. Hajian et al. [25] suggested that roflumilast may enhance the efficacy of ICS/LABA by reducing inflammation and edema via opening smaller airways or preventing airway collapse, thereby reducing regional overinflation. In a receiving appropriate combination therapy (REACT) trial, roflumilast in combination with ICS/LABA significantly reduced rates of exacerbation and hospitalization in moderate to severe COPD [10], which was consistent with our results.

More AEs and higher AE incidence were observed in the roflumilast group than the placebo group. In previously pooled analyses, this therapy mainly affects the gastrointestinal tract and nervous system, and the most common AEs comprise diarrhea, nausea, headache, and weight loss [9, 28], which are empirical PDE4 inhibitor-associated AEs [29]. And the incidence of this therapy is in accordance with that of a previous 6-month RCT of roflumilast [30]. In this study, compared with patients taking placebo, the most reported AEs were decreased appetite and weight loss in those taking roflumilast. And patients in the roflumilast group are elucidated to lost more weight [10, 17]. Among adverse reactions, pneumonia was proved to be correlated with an increased risk of death in COPD [31], and the use of ICS leads to an increased risk of pneumonia in COPD patients [32]. Roflumilast was not explored to increase the incidence of pneumonia in our study (*P* = 0.85). During the study, approximately 2%-3% of patients died mainly due to COPD exacerbation and AEs [10], with no difference in mortality between the roflumilast and placebo groups (*P* = 0.74).

However, several limitations existed in this study. First, little literature containing RCTs was included, whose results might not fully reflect the treatment situation. Second, various patients in the roflumilast group quit the trial due to AEs than those in the control group, which did not indicate the true incidence of AEs. Third, confined to the data provided by the original study authors, this study was unable to conduct a subgroup analysis, and expanded studies are needed in the future to characterize the population with the greatest benefit from this therapy. Finally, the evaluation of publication bias and funnel plot was not carried out in this study because less than 10 literatures were included.

Taken all together, according to the completed RCTs, roflumilast was dramatically effective to patients with severe and profound COPD treated with ICS/LABA and notably reduced the incidence of exacerbation but brought PDE4 inhibitor-associated AEs.

## Figures and Tables

**Figure 1:** Flow chart of literature screening process.

**Figure 2:** The quality assessment of the included literature: (a) overall bias risk; (b) bias risk for each RCT.

**Figure 3:** Comparison of FEV_1_ changes before bronchodilator administration between the roflumilast group and placebo group.

**Figure 4:** Comparison of FEV_1_ changes after bronchodilator administration between the roflumilast group and placebo group.

**Figure 5:** Comparison of COPD exacerbation rate between the roflumilast group and placebo group.

**Figure 6:** Comparison of incidence of adverse reactions between the roflumilast group and placebo group.

**Figure 7:** Comparison of incidence of adverse reactions between the roflumilast group and placebo group (no difference).

**Table 1:** Primary characteristics of the eligible studies in more detail.

Author (year)	Phase	No. of patients		Male, *n* (%)		Age, mean (SD)		COPD severity, *n* (%)			
								Severe		Very severe	
		Roflumilast	Placebo	Roflumilast	Placebo	Roflumilast	Placebo	Roflumilast	Placebo	Roflumilast	Placebo
Calverley PM (2007)	IV	1,178	1,174	821 (70)	794 (68)	64 (8.8)	65 (8.4)	508 (67)	510 (68)	181 (24)	176 (23)
Calverley PM (2009)	IV	973	972	718 (74)	725 (75)	65 (8.4)	65 (8.4)	943 (61)	989 (64)	463 (30)	440 (28)
Rennard SI (2011)	IV	30	11	NR	NR	64 (7.4)	70 (6.8)	356 (63)	399 (66)	148 (26)	169 (28)
De Backer W (2014)	III	567	606	387 (68)	400 (66)	64 (8.7)	64 (8.8)	NR	NR	NR	NR
Martinez FJ (2015)	III	1,537	1,154	1,150 (75)	1,186 (76)	64 (9.0)	64 (9.0)	678 (70)	677 (70)	291 (30)	273 (28)
Martinez FJ (2016)	III	760	753	571 (75)	574 (76)	65 (9.6)	64 (9.1)	698 (59)	720 (61)	474 (40)	446 (38)

NR: no report.

## Data Availability

No additional data are available.
